The article "Multiagent Culture Algorithm-Based Interactive Design of College English Online Teaching Process" was retracted in 2023. Reasons: unreliable results or conclusions; concerns about the data; concerns about the peer review; concerns about the citations.

# Multiagent Culture Algorithm-Based Interactive Design of College English Online Teaching Process

**DOI:** 10.1155/2022/3490055

**Published:** 2022-05-31

**Authors:** Nianfan Peng

**Affiliations:** School of Foreign Studies, Guangzhou University, Guangzhou, Guangdong Province, China

## Abstract

Traditional educational techniques and conceptions no longer match the need of the society for talent training. It is due to the fact that educational reforms are deepening and more open interactive teaching models have begun to be gradually implemented in college English instruction. The method's innovation and reform can not only fully respect the students' dominating position but also entice students to devote themselves to the English classroom with greater zeal which is helpful in allowing for deeper knowledge discovery and thinking. This study has the motive to examine the interactive teaching mode's application tactics in college English classrooms, particularly with the goal of improving the effectiveness of English classroom teaching and promoting the high-quality growth of today's college students. Furthermore, in order to improve the interactivity of online English teaching in colleges and universities, this research proposes an intelligent conversation system based on multiagents to aid in the improvement of online teaching. Finally, using a public discourse corpus dataset for implementation, the proposed model proves to have better performance than existing state of the art approaches.

## 1. Introduction

In today's world, English is the worldwide language of globalization and it holds a prominent role in the country's educational system especially China. However, despite the fact that the kids have been receiving English instruction for more than ten years, their learning effect has not reached the level that was anticipated. None of them is able to communicate and read in English fluently on a regular basis. Specifically, this is due to the fact that the primary form of instruction for English education in our country is indoctrination [1–4]. The process of students learning English is the process of mechanically memorizing words and grammar, which not only reduces students' interest in learning to a significant extent but also causes English to lose its practicality so that it no longer exists as a language of communication, but rather as a subject for examination. Students' core literacy education must be nurtured, which means that college English teaching must undergo innovative reforms, adopt more diversified teaching modes in order to further improve the teaching efficiency of English subjects, and promote the overall improvement of college students' English quality [5, 6].

The article "Multiagent Culture Algorithm-Based Interactive Design of College English Online Teaching Process" was retracted in 2023. Reasons: unreliable results or conclusions; concerns about the data; concerns about the peer review; concerns about the citations.

The multidimensional interactive teaching mode that emerged against the backdrop of information technology has played a significant role in the development of high-level talents in the new era, and as a result, it is widely used in classroom teaching at major colleges and universities across the country [7, 8]. The level of social competition that now exists is extremely high. Effective implementation of a multidimensional interactive teaching mode especially in college classroom instruction will not only assist college students to improve their learning and communication skills, but it will also assist them in improving subjective initiative and professional level. Apart from it, it will also help them in obtaining their own competitive bargaining chips. However, there are still a number of shortcomings and flaws in the implementation of the multidimensional interactive teaching mode in English instruction in various colleges and universities, which have an adverse influence on the effectiveness of the mode's application. For this reason, the study addresses the method for optimizing the implementation of multidimensional interactive teaching mode in the context of college English instruction [9, 10].

Interaction is defined as the process of interaction between individuals or groups and between groups. When it comes to education, interaction serves the function of a medium of exchange that can support the further expansion of the form and content of instruction. It is also based on the traditional educational model, which is why it has been introduced in this field. This is a new concept. Interaction can help to strengthen the bond that exists between teachers and students, as well as to innovate teaching methods, expand teaching content, and make learning more engaging in the classroom [11–15]. Using a multidimensional interactive teaching model, teachers are responsible for regaining control of the classroom by focusing on the actual development needs of students, organizing and leading teaching activities around curriculum knowledge, creating interactive links between teachers and students, and ensuring that students are participating in the learning activities. Teachers are responsible for ensuring that students are participating in the learning activities. It is possible to harvest.

As a result of the rapid expansion of society and the economy, my country has experienced an increase in the frequency of global economic and trade transactions, and the demand for high-quality English abilities has increased in tandem. Students can be supplied with an oral communication platform through the use of a multidimensional interactive teaching mode in English classes at colleges and universities, as well as other educational institutions. It has been demonstrated that students' knowledge application ability has increased under the leadership of teachers, as well as that students' passion and enthusiasm may be stimulated to assist them in forming English literacy and continuing to progress. developing [16, 17].

The article "Multiagent Culture Algorithm-Based Interactive Design of College English Online Teaching Process" was retracted in 2023. Reasons: unreliable results or conclusions; concerns about the data; concerns about the peer review; concerns about the citations.

There have also been numerous studies on neural task dialogue systems that have sprung up as a result of the advancement of deep learning. It is divided into four sections: Natural Language Understanding (NLU), Dialog State Tracking (DST), Dialog Policy Learning (DPL), and Natural Language Generating (NLG) [18–24]. The conversation strategy, for example, is responsible for selecting the next action to be performed in accordance with the existing condition, and it plays a significant part in the task dialogue system. The overall system's performance is directly influenced by the quality of the data. Because of its Markov nature, it is frequently referred to as a reinforcement-learning problem, in which users are portrayed as being a part of the environment and policies are learned by interaction with the users. Given that reinforcement learning demands a significant amount of interactivity throughout the training process, it takes a significant amount of time and money to connect with real users. The training of a user simulator with human dialogue data is one way that might be used. This would allow the system agent to learn dialogue policies through interaction with the user simulator. In addition, the simulator may be used to replicate human behavior in offline settings at no additional expense, and the trained system can subsequently be deployed and fine-tuned by interacting with real users. Making a trustworthy user simulator, on the other hand, is not an easy or without its difficulties. Because of the increasing variety of business scenarios and the increasing complexity of task functional requirements, developing a completely rule-based user simulator will require a significant amount of multidomain expertise, which will be a difficult undertaking. Recently, several academics have proposed data-driven user simulators in light of the advancement of machine learning; however, this requires a large amount of manually annotated data, which is not readily available [25–31].

This paper proposes an interactive method for the college English online teaching process that is based on a multiagent cultural algorithm. In order to address the challenge of generating a reliable user simulators for dialogue strategy learning as well as to improve the interactivity of college English online teaching. It first learns directly from the dialogue corpus while being trained in imitation learning under supervision and then uses this knowledge to drive the policies of both the basic system and user agents, respectively. In the following step, the task-oriented interactive discussion between the two agents is simulated, and the reinforcement-learning algorithm optimizes its dialogue approach in order to further improve the performance of the system. At the end of the study, the relevant performance is assessed using the MultiwOz101 task-oriented multidomain multi-intent discourse corpus.

The article "Multiagent Culture Algorithm-Based Interactive Design of College English Online Teaching Process" was retracted in 2023. Reasons: unreliable results or conclusions; concerns about the data; concerns about the peer review; concerns about the citations.

The rest of the manuscript is arranged according to the following agenda items.

A comprehensive review of the existing literature is presented in section background. The interactive method for the college English online teaching process that is based on a multiagent cultural algorithm is described in detail in section entitled as method. Results of the proposed scheme in terms of various performance evaluation metrics are compared and reported in the results section. Finally, concluding remarks are given at the end in the form of an extensive summary.

## 2. Background

### 2.1. Current Situation of English Teaching

#### 2.1.1. Single Teaching Mode

Students' primary motivation for learning English in college and university settings is to pass the CET-4 and CET-6 tests, which is a compelling reason to learn the language. As a result, during the course of the instructional process, teachers will pay close attention to the pursuit of students' test scores and pass rates. Make English a test topic rather than a practical language subject by making it an exam subject. In spite of the fact that various new teaching concepts and teaching methods continue to flood the market as a result of the ongoing deepening of education reform, some English classes are still taught by teachers, and students are accepted mechanically in order to improve the passing rate in colleges and universities. Students appear to have strong written test scores, but their listening and communication abilities are often lacking, which is referred to as a dumb English problem in this context. In addition, some English teachers fail to consider the spiritual development of their pupils when imparting English information, and they do not engage in cross-cultural educational activities. For student, the goal of English language teaching and learning is to improve their ability to communicate effectively in a globalized environment. In addition to the foreign language tuition and cultural knowledge, cultivating students' self-confidence in Chinese culture and putting our own excellent teaching and learning practices into practice. Spread things out, be able to tell Chinese stories well, possess qualifications as a qualified cultural communicator. Finally, they must be capable of effectively and accurately using English as a foreign language in an intercultural and multicultural environment are all requirements for me to make use of the language.

The article "Multiagent Culture Algorithm-Based Interactive Design of College English Online Teaching Process" was retracted in 2023. Reasons: unreliable results or conclusions; concerns about the data; concerns about the peer review; concerns about the citations.

#### 2.1.2. Failure to Fully Respect the Dominant Position of Students

Despite the fact that the reform of quality education has been in full motion for quite some time, the influence of exam-oriented education continues to be difficult to erase. When it comes to learning English, many college students have set their learning thoughts and learning practices in stone. Despite the fact that many college students have excellent results in CET-4 and CET-6, the application system for English is not complete; it is simple to pass the test, but more difficult to apply and communicate once you have passed. Consequently, many college students struggle to simply identify themselves fluently after graduation, and their vocabulary mastery has not significantly increased when compared to that of middle-school pupils. This is primarily due to the fact that teachers do not fully respect students' dominant position in the teaching process, do not recognize the purpose of English communication, and do not interact effectively with students during the teaching process, resulting in a lack of practical exercises in the language learning process and college students being unable to rely on interest for autonomy. Learning can only be done for the sake of learning, which contributes to the fact that most college students lack fluent English conversation skills as well as practical application abilities.

### 2.2. Interactive Teaching Strategies

#### 2.2.1. Diversified Teaching Methods

Teachers must use a variety of teaching methods in the classroom in order to further improve the applicability of talents. They must also be able to combine the individual differences of students in order to teach students according to their aptitude in order to truly maximize the value of the interactive teaching mode. Using the so-called “interactive teaching” style in the English classroom, teachers can provide students additional opportunities to communicate with one another, allowing them to practice their English abilities in real-life circumstances. However, because college students have varying levels of English proficiency, if teachers are unable to teach students according to their aptitude but instead arrange unified discussion topics, some students will be conflicted because they do not understand, and some students will be too simple and lose exploration. desire. The teachers' capacity to use a range of teaching methods, correctly recognize and comprehend the differences between students, and teach students according to their aptitude in the teaching process are all necessary to further increase the practicability of an interactive teaching model [32, 33].

The article "Multiagent Culture Algorithm-Based Interactive Design of College English Online Teaching Process" was retracted in 2023. Reasons: unreliable results or conclusions; concerns about the data; concerns about the peer review; concerns about the citations.

Teachers, for example, use a hierarchical teaching style to help students learn more effectively. During the teaching process, college English teachers can combine students' actual learning ability with comprehensive English quality, divide students into different levels, and formulate different learning methods and learning goals for each level, allowing each student to be at his or her own level. Obtain the greatest possible development of talent and continue to rise to greater levels of achievement. Students' enthusiasm in studying is increased, and their English proficiency is consistently improved, as a result of step-by-step encouragement and support from the instructor. For example, when teachers guide students through the writing process, they can assign different writing tasks to students at various levels of proficiency. When students are assigned to work on Ren Nu, they are allowed to discuss the writing assignments, sort out their writing ideas, and develop their oral expression and organizing abilities. Finally, they should sort out their own viewpoints and produce an outstanding piece of written work in English.

Additionally, the group cooperative teaching approach has become increasingly popular in English education at both the college and university levels. It is possible for teachers to separate students into different groups and encourage students to participate in group discussions about course topics. If, for example, English teachers explain the reading lesson, they can provide discussion themes to encourage students to explore the content of the text in English and ask specific questions. During the conversation, teachers should also provide appropriate assistance to students in order to help them organize their thoughts and construct the knowledge framework of the book. Students can also engage in debates on other points of view in order to further develop their interpersonal and communication abilities. It is possible to create a more relaxed conversation atmosphere in this group cooperative teaching style, and throughout the discussion, teachers can gain a specific grasp of the students' learning situation, allowing them to provide focused explanations in the following teaching process. The group cooperative teaching mode can also help college students develop their team consciousness and cooperation consciousness, which can aid them in developing their strengths and avoiding their shortcomings, as well as assisting them in achieving the common progress of all students [34].

The article "Multiagent Culture Algorithm-Based Interactive Design of College English Online Teaching Process" was retracted in 2023. Reasons: unreliable results or conclusions; concerns about the data; concerns about the peer review; concerns about the citations.

#### 2.2.2. Utilize Modern Teaching Methods

Modern English teachers should make full use of modern teaching methods in the classroom in order to create a more efficient and dynamic learning environment for their pupils, especially in light of the ongoing advancement of information technology. Using microlecture videos, teachers can create flipped classrooms for their students, effectively transforming typical indoctrination classrooms into inquiry-based learning environments. Specific to teaching content, teachers must prepare lessons in a scientific manner for students to learn, clarify teaching ideas and key points, and record student micro-lecture videos, which are send to students on a public learning platform before class so that students can preview independently and identify problems before they occur. During the formal teaching period, the teacher should give targeted explanations based on the students' questions in order to help the students understand both important and difficult teaching points in this class. You can also feedback questions that appeared in the preview on the learning platform, as well as communicate with the students through the learning platform; Increase the clarity of your corpus of knowledge. The teachers' focus should be on creating a more relaxed communication environment for students during the explanation process, so that students can engage in bold discussions about important and difficult teaching points and put forward innovative opinions and insights, cultivate students' creative thinking, and encourage students to think critically and creatively about their learning. For self-directed learning after class, students should review the microclass resources several times in order to internalize and absorb classroom knowledge, as well as interact and discuss with other students in the message area, in order to truly transform book knowledge into practical application ability and achieve comprehensive improvement in their English language proficiency.

#### 2.2.3. Arouse Students' Interest

Students' willingness to participate in the classroom and their desire to learn can both be increased through interaction in the interactive teaching method, which is one of its most important characteristics. For this reason, English teachers must be familiar with the psychological characteristics of contemporary college students, as well as be able to grasp a general understanding of their interests and concerns, in order to more effectively locate the entry point of the classroom and more effectively attract college students' attention in the English classroom. College students today are a flamboyant breed of individuals with strong personalities. They each have their own unique set of thoughts and opinions on a wide range of topics. Teachers can make full use of their personal characteristics and combine the content of teaching materials to transform classrooms into debate venues, small theaters, and other simulated activities for students, as well as to transform classrooms into debate venues, small theaters, and other simulated activities. Due to the circumstances, students are more likely to engage in in-depth conversations and exchanges about the course material. In the case of a textbook, teachers can create a script outlining the topic and then use the script to pique the interest of students in the subject matter. They can then urge students to role-play in the classroom.

The article "Multiagent Culture Algorithm-Based Interactive Design of College English Online Teaching Process" was retracted in 2023. Reasons: unreliable results or conclusions; concerns about the data; concerns about the peer review; concerns about the citations.

Students are obligated to rehearse their lines on a regular basis. At the same time, students can converse and communicate in English in a real environment, allowing them to truly experience the allure of the English language. Apart from that, teachers can make full use of multimedia and other teaching equipment, locate some classic English videos, encourage students to dub them, and hold dubbing competitions to enrich students' English classrooms and create a more relaxed and enjoyable learning environment for students. Encourage pupils to develop into innovative talents with a broad range of abilities in order to fully realize their independence in learning. Additionally, English teachers in colleges and universities should strive to provide as many English communication platforms for college students as possible, allowing them to have a better understanding of the importance of English in a real-world communication environment. When teaching English in a classroom context, English teachers can blend students' majors together. Specific English circumstances, such as commercial discussions and economic transactions, that students will encounter after graduation provides students with the opportunity to practice their language abilities in realistic situations and put what they have learned to good use immediately.

Teachers should continue to use various resources to enrich teaching materials during the teaching process in order to further stimulate students' interest in learning. They should also fully explore the differences between Chinese and Western cultures in the teaching materials in order for students to correctly understand and understand both Chinese and Western cultures. The cultural background and logical connotation of textbook articles should be explained as well, so that students can understand the main points of the articles more deeply on the basis of understanding their literal meaning, avoid students from forming knowledge gaps, and achieve language knowledge and cultural connotations as part of the process of explaining the textbook articles. Maintain a healthy balance, and assist students in developing a more methodical English thinking system in order to consistently improve their communication skills in English.

The article "Multiagent Culture Algorithm-Based Interactive Design of College English Online Teaching Process" was retracted in 2023. Reasons: unreliable results or conclusions; concerns about the data; concerns about the peer review; concerns about the citations.

## 3. Method

The goal of this work is to learn multiagent dialogue policies in task dialogue systems, which will be used in future work. The user agent and the system agent communicate with one another in order to achieve the user goal, and the system agent consults an external database in order to deliver entity information to the user as needed.

User goal *G*=(*R*, *C*) consists of user constraint *C* and a request *R*, *G* is known only to the user agent, external database DB contains all entities and related information, and only system agents can access the DB. If there are multiple domains in *G*, two agents need to complete subtasks in each domain. In a single dialogue round, the user agent first initiates a query request, and then the system agent replies with a response, and the two are executed alternately. Therefore, each dialogue *τ* can be viewed as a sequence of state-action pairs, which are as follows:

(1) $$\begin{array}{c} \left\{\left(s_{0}^{U},a_{0}^{U},s_{0}^{S},a_{0}^{S}\right),\left(s_{1}^{U},a_{1}^{U},s_{1}^{S},a_{1}^{S}\right),\cdots \right\}, \end{array}$$

where the user agent and the system agents make decisions according to their respective policies *μ*(*a*^*U*^∣*s*^*U*^), *π*(*a*^*S*^∣*s*^*S*^). The model proposed in this paper is shown in Figure 1.

The dialogue state *s* of the system agent in the *t*-th round consists of six parts:

1. The user action *a*_*t*_^*U*^ of the current round.
2. The system action *a*_*t*−1_^*S*^ of the previous round.
3. The confidence of the current round state _*b*_^*t*^, used to track the constraints and request information provided by the user agent.
4. The entity result *q*_*t*_ queried from the external database DB.
5. The domain information *d* predetermined by the system.
6. The terminal signal of whether the dialogue ends *T* ∈ {0,1}.

In order to avoid obtaining reward returns that may cause high variance when sampling the entire trajectory, this paper directly uses the estimated cumulative reward for optimization, takes full advantage of the Actor–Critic method, and performs training under the CTDE architecture. The calculation formula is as follows:

(2) $$\begin{array}{c} V\left(s_{t}\right)=E\left|R_{t}\right|=E\left|\sum_{lk=\geq t}\gamma^{l-t}r_{t}\right|. \end{array}$$

As shown in Figure 2, this paper designs a user-system mixed value evaluation network with soft attention state sharing by using the sigmoid function on the encoding vector for the evaluation of related values. The design of this soft attention mechanism refers to Reference [12]. Specifically, the user agent state *s*^*U*^ and the system agent state *s*^*S*^ are first calculated through a soft attention layer to obtain the respective encoded information vectors *h*^*U*^ and *h*^*S*^. The formula is as follows:

(3) $$\begin{array}{c} h^{U}=\sigma \left(f_{1}^{U}\left(s^{U}\right)\right)⊙\;\tanh\left(f_{2}^{U}\left(s^{U}\right)\right),\\ h^{S}=\sigma \left(f_{1}^{S}\left(s^{S}\right)\right)⊙\;\tanh\left(f_{2}^{S}\left(s^{S}\right)\right). \end{array}$$

The calculation formula of the fusion information vector *h*^*G*^ is as follows:

(4) $$\begin{array}{c} h^{G}=\frac{1}{\left|V\right|}\sum_{v\in \left\{U,S\right\}}h^{v}+\text{Max}\left(h^{U},h^{S}\right). \end{array}$$

Finally, pass the obtained *h*^*U*^, *h*^*S*^, and *h*^*G*^ to the specific task layer to obtain the final values *V*^*U*^, *V*^*S*^, and *V*^*G*^:

(5) $$\begin{array}{c} V^{U}=f^{U}\left(h^{U}\right),\\ V^{S}=f^{S}\left(h^{S}\right),\\ V^{G}=f^{G}\left(h^{G}\right). \end{array}$$

When dealing with multidomain, complex dialogue jobs, the action space of policies can grow extremely enormous, making it nearly impossible to explore and learn dialogue policies from the ground up from the beginning. As a result, this paper first optimizes using imitation learning-behavioral cloning before moving on to the next step.

The article "Multiagent Culture Algorithm-Based Interactive Design of College English Online Teaching Process" was retracted in 2023. Reasons: unreliable results or conclusions; concerns about the data; concerns about the peer review; concerns about the citations.

In the first step, the state-action pair is extracted from the dialogue trajectory of real human dialogue data, and the state is regarded as an input feature and the action is regarded as an output tag for classification and learning. After that, the optimal policy model is obtained by combining the state and action pairs. The logistic regression method is used in this research for policy pretraining. Furthermore, because a single agent may only provide a finite number of dialogue behaviors in a dialogue round, *α* weights are applied to the labels in order to lessen the bias of the data, and the loss function is defined as follows:

(6) $$\begin{array}{c} L\left(x,y;\alpha \right)=-\alpha \cdot Y^{T}\log\;\sigma \left(x\right)-\left(1-Y^{T}\right)\log\left(1-\sigma \left(x\right)\right). \end{array}$$

PPO is the second optimization stage, and it is consistent with other research in the field. The GAE algorithm, in particular, is used by the advantage function to balance the bias and variance of the Critic, among other things. The GAE estimators that were employed were as follows:

(7) $$\begin{array}{c} {\hat{A}}_{t}=\omega_{t}+\gamma \lambda {\hat{A}}_{t+1},\\ \omega_{t}=r_{t}+\gamma V_{\theta }\left(s_{t+1}\right)-V_{\theta }\left(s_{t}\right). \end{array}$$

The article "Multiagent Culture Algorithm-Based Interactive Design of College English Online Teaching Process" was retracted in 2023. Reasons: unreliable results or conclusions; concerns about the data; concerns about the peer review; concerns about the citations.

## 4. Results

Specifically, MutiWOZ is used in this paper, which is a task-oriented multidomain multi-intent conversation corpus consisting of seven domains, thirteen intentions, ten thousand eight hundred and forty-three dialogues, and seven hundred and forty-four dialogue turns. User goals are established before to data collection, and users are given the option to adjust their goals during the interaction. As a result, the data obtained is more representative of real-world discussions than the data collected during data collection. Ontologies are also provided by the corpus, which defines all of the entity properties of the external database.

The most important evaluation factors are the expense of the dialogue and whether or not the dialogue task has been fulfilled. It is calculated in this study that the number of dialogue turns (DT), task success (TS), Inform F1 (IF), and Matchrate (MR) all contribute to the cost of dialogue. The algorithms used in this research for comparison include SL, RL, and TRPO.

TS, IF, and MR indicators are shown in Figure 3 in the context of comparative experimental results for TS, IF, and MR indicators, where the strategies of the user agent and the system agent are trained in response to specific conditions. It can be noted that, when compared to the other models in the picture, the performance of the model described in this work has significantly increased, with task success reaching 84.5%, a value that is 15.2% higher than the TRPO model.

Figure 4 shows a comparison of the number of dialogue turns required for various strategies. The model performs best when the number of turns is kept to a minimum.

As can be seen in Figure 4, the number of dialogue rounds required by the model in this research is 6.13, and the dialogue cost is the lowest of the models considered. The following are the reasons we believe this is the case: first, on the basis of imitation learning, the two agents are further trained by reinforcement learning, which reduces the amount of time spent training and increases the efficiency of the training process. Second, in a dynamic environment, the two agents alternate training at the same time, allowing them to adapt to a variety of different situations. The value estimate learned by the user-system hybrid value assessment network using soft attention state sharing can also be used to better guide the updating of policy gradients.

The article "Multiagent Culture Algorithm-Based Interactive Design of College English Online Teaching Process" was retracted in 2023. Reasons: unreliable results or conclusions; concerns about the data; concerns about the peer review; concerns about the citations.

Further, we conduct ablation experiments on the DT metric. We first removed soft attention (SA), and PPO, respectively, and then removed SA and PPO at the same time, and finally calculated their respective DT values, as shown in Figure 5.

It can be seen from Figure 5 that the effect of removing PPO on the model is greater than removing SA, and removing PPO and SA at the same time has the greatest impact.

## 5. Conclusion

Traditional education techniques and educational conceptions no longer suit the needs of society in terms of talent promotion, and more open interactive teaching modes are gradually being implemented in English courses at colleges and universities as part of the education reform process. Essentially, this is a reinterpretation and revision of the classic indoctrination instructional approach. A specific analysis is conducted in this paper on how to implement a strategy of interactive teaching mode in a college English classroom in order to continuously improve the effectiveness of English classroom instruction while also promoting the high-quality growth of contemporary college students. Furthermore, in order to improve the interactivity of online English teaching in colleges and universities, this study proposes an intelligent conversation system based on multiple intelligences, which can be used to enhance the online English teaching process in colleges and universities. Finally, the performance of the algorithm is evaluated using a publicly available conversational corpus dataset, which is presented in this study.

## Figures and Tables

**Figure 1:** The structure of the multiagent dialogue system.

**Figure 2:** The structure of the Critic Network.

**Figure 3:** Comparison of TS, IF, and MR on the MultiWOZ dataset.

**Figure 4:** Comparison of DT on the MultiWOZ dataset.

**Figure 5:** Ablation experiment results.

## Data Availability

The data used to support the findings of this study are available from the corresponding author upon request.
